# Role of T follicular helper cells and their associated molecules in the pathogenesis of chronic hepatitis B virus infection

**DOI:** 10.3892/etm.2012.864

**Published:** 2012-12-19

**Authors:** TONGJING XING, HONGTAO XU, WENQING YU

**Affiliations:** Department of Infectious Diseases, Taizhou People’s Hospital, Taizhou, Jiangsu 225300, P.R. China

**Keywords:** T follicular helper cells, interleukin-21, chronic hepatitis B

## Abstract

In this study, we investigated the roles of T follicular helper (TFH) cells and related molecules in the pathogenesis of chronic hepatitis B virus (HBV) infection. The levels of circulating TFH cells and their surface CD40 ligand (CD40L), as well as CD19^+^ B cells and their surface CD40 expression were detected by flow cytometry. Peripheral blood plasma interleukin (IL)-21 levels were detected by enzyme-linked immunosorbent assay (ELISA). Compared with hepatitis B surface antibody (HBsAb)^−^ and HBsAb^+^ healthy controls, the percentage of TFH cells and their surface CD40L expression significantly increased in patients with chronic HBV infection, particularly those with chronic hepatitis B (P<0.05). The percentage of CD19^+^ B cells significantly increased in chronic hepatitis B patients and CD40 expression levels on the CD19^+^ B cell surface in chronic HBV infection decreased compared with those in the healthy controls (P<0.05). Compared with the healthy controls, the plasma IL-21 level in chronic hepatitis B patients was significantly increased in chronic HBV carriers and decreased in inactive hepatitis B surface antigen (HBsAg) carriers (P<0.05). The TFH cell percentage, B cell percentage and IL-21 expression did not significantly differ between the hepatitis B e-antigen (HBeAg)^−^ and HBeAg^+^ chronic hepatitis B groups (P>0.05). The abnormal expression of TFH cells and IL-21 is related to the dysfunction of immune response during chronic HBV infection. The interaction of CD19^+^ B cells with TFH cells via their CD40 and CD40L molecules may also play an important role in this process.

## Introduction

Chronic hepatitis B (CHB) is an infectious disease that severely harms individuals worldwide. Although new cases of hepatitis B virus (HBV) infection are greatly reduced by the application of a hepatitis B vaccine, >350 million individuals are infected with HBV worldwide. Persistent HBV infection may lead to cirrhosis or hepatocellular carcinoma, which threaten the lives of patients (1). Virus-host interactions, particularly the virus-specific T-cell response, are the key factors accounting for the pathogenesis of HBV infection. In contrast to the strong and multispecific T-cell responses observed during acute self-limited HBV infection, patients with CHB tend to have weak and narrowly focused immune responses (2).

CD4^+^ T cells play a vital role in adaptive immune responses. They help B cells produce antibodies and undergo class-switching, as well as affinity maturation. They recruit and activate CD8^+^ T cells, macrophages and other effector cells. T helper cells, differentiated from naive CD4^+^ T cells, are classified into four major lineages based on their function, pattern of cytokine secretion and expression of specific transcription factors. The lineages are Th1, Th2, Th17 and T regulatory cells (3,4). The assistance of antibody production by T cells is a fundamental aspect of immune responses. An improved understanding of the cellular and molecular mechanisms of T cell actions has only recently emerged. A subset of T cells named T follicular helper cells (TFH cells) aid B cells and represents one of the largest and most important subsets of effector T cells in lymphoid tissues (5,6). The features of TFH cells include CXC chemokine receptor 5 (CXCR5) expression, inducible co-stimulator (ICOS), location/migration (B cell follicles) and function (B cell help). TFH cells produce a ‘helper’ cytokine, interleukin (IL)-21, which stimulates B cells to differentiate into antibody-forming cells via the IL-21 receptor. The dysregulation of TFH cell function likely contributes to the pathogenesis of immune-related diseases (7).

Humoural immune responses following HBV infection are significant in the pathogenesis of HBV infection. Hepatitis B surface antigen (HBsAg)-specific antibodies neutralise and mediate protective immunity. HBV-specific antibodies are indicators of specific stages of the disease. Hepatitis B core antigen (HBcAg)-specific immunoglobulin G (IgG) and HBsAg-specific antibodies persist for life following clinical recovery (8). TFH cells are a special subset of T helper cells that regulate humoural immune responses. However, the role of TFH cells in the pathogenesis of HBV infection is unclear. Therefore, in the present study, the levels of TFH cells and related molecules were detected in various types of chronic HBV infection by flow cytometry and enzyme-linked immunosorbent assay (ELISA). The purpose was to investigate the role of TFH cells and related molecules in the pathogenesis of CHB.

## Materials and methods

### Subjects

Blood samples were obtained with informed consent from 85 patients infected with HBV and 44 healthy controls at the Taizhou People’s Hospital from June to December 2011. There were 42 patients with CHB (male to female ratio, 29:13; average age, 40.7±11.2 years) and 43 HBV carriers (male to female ratio, 28:15; average age, 41.3±11.6 years). Of the 42 patients with CHB, 18 hepatitis B extracellular antigen (HBeAg)^+^ patients and 24 HBeAg^−^ patients were included. Of the 43 HBV carriers, 21 chronic HBV carriers and 22 inactive HBsAg carriers were included. The protocol was approved by the ethics committee of the hospital. The diagnostic criteria were based on the 2010 Chronic Hepatitis B Prevention Guide of China (9). All patients tested negative for antibodies against hepatitis A, C, D and E viruses, as well as human immunodeficiency virus. Patients with a history and clinical features of drug-induced liver injury, alcoholic hepatitis and steatohepatitis were also excluded. Any patients who had been treated with nucleoside/nucleotide analog antiviral or immunomodulatory drugs in the previous six months were excluded. There were 22 cases that were hepatitis B surface antibody (HBsAb)^+^ following inoculation with a hepatitis B vaccine (male to female ratio, 13:9; average age, 38.7±10.3 years) and 22 HBsAb^−^ cases who had not been inoculated with a hepatitis B vaccine (male to female ratio, 10:12; average age, 40.5±10.6 years) included as healthy controls. Subjects who were HBeAb^−^ and/or HBcAb^+^ were excluded.

### Flow cytometry analysis

Sodium citrate-treated whole blood (100 *μ*l) was added to 10 *μ*l Alexa Fluor 647-conjugated anti-CXCR5 (BD Company, San Jose, CA, USA) and 10 *μ*l fluorescein isothiocyanate (FITC)-conjugated anti-CD4 (eBioscience, San Diego, CA, USA), then mixed and incubated for 30 min at room temperature. Erythrocytes were lysed by adding 2 ml fluorescence-activated cell sorting (FACS) lysing solution. The samples were analyzed on a FACS cytometer using CellQuest™ software (Fig. 1). CD40L-PE/CD40-PE and CD19-FITC were purchased from eBioscience. The expression of CD40L on the surface of TFH cells and CD40 on the surface of CD19^+^ B cells were detected as described above.

### Cytokine detection

The level of IL-21 in stored peripheral plasma was evaluated by ELISA. The kits were purchased from eBioscience and used according to the manufacturer’s instructions. The detection range for IL-21 in this kit was 16-2000 ng/l.

### Detection of HBV DNA and serum markers

The levels of HBV DNA were detected by fluorescence quantitative polymerase chain reaction (PCR; lower detection limit, 10^3^ copies/ml; Applied Biosystems, Foster City, CA, USA). HBV PCR fluorescence quantitative detection kits were purchased from Biological Engineering Co., Ltd. (Shanghai, China). The serum markers of HBV, anti-HAV, anti-HCV, anti-HDV and anti-HEV, were detected by ELISA. The kits were purchased from Beijing Yuanpinghao Biotechnology Co., Ltd. (Beijing, China).

### Statistical analysis

All values are expressed as the median and quartile interval. Data analysis was conducted using SPSS 17.0 (SPSS Inc., Chicago, IL, USA). Nonparametric tests (Kruskal-Wallis H test) were used for multiple group comparison. The Mann-Whitney U test was used for two independent data. The Spearman correlation was used between variables. P<0.05 was considered to indicate a statistically significant difference.

## Results

### Proportion of TFH cells and levels of CD40L expression on the surface of TFH cells

The proportion of TFH cells gated with CD4^+^ T cells and CD40L expression level were detected by flow cytometry in 42 patients with CHB, 43 HBV carriers and 44 healthy controls. Compared with the HBsAb^−^ and HBsAb^+^ healthy controls, patients with chronic HBV infection had significantly increased percentages of TFH cells (P<0.01). The percentage of TFH cells was higher in the patients with CHB than in the chronic HBV carriers (P<0.01). The percentage of CD40L in chronic HBV infected individuals was significantly higher than in the HBsAb^−^ and HBsAb^+^ healthy controls (P<0.01). The pattern of coexpression of CXCR5 and CD40L in the CD4^+^ T cells in the different groups was similar to that of the TFH cells. No significant difference was observed in the percentage of TFH cells or CD40L between the HBsAb^−^ and HBsAb^+^ healthy controls (Fig. 2).

### Detection of the expression of CD19^+^ B cells and their surface CD40 molecules in different subjects

The percentage of CD19^+^ B cells and their surface CD40 molecule expression were detected by flow cytometry in different subjects. Compared with the HBsAb^−^ and HBsAb^+^ healthy controls, the percentage of CD19^+^ B cells in patients with CHB increased significantly (P<0.05). No significant difference was observed between chronic HBV carriers and inactive HBsAg carriers (P>0.05). The percentage of CD40 molecules on the surface of CD19^+^ B cells in the CHB patients was lower than that in the HBsAb^−^ healthy controls (P<0.01). No significant difference was observed among the remaining groups (P>0.05; Fig. 3).

### Detection of plasma IL-21 expression in different subjects

The plasma IL-21 expression level in the different subjects was detected by ELISA. Compared with the HBsAb^−^ and HBsAb^+^ healthy controls (332.7±202.5 and 295.3±108.6 ng/l), plasma IL-21 expression was markedly decreased in the HBV carriers and inactive HBsAg carriers (239.6±195.9 and 215.5±132.0 ng/l, respectively; P<0.05). However, plasma IL-21 expression in the CHB patients (375.6±192.3 ng/l) was significantly higher than that in the HBsAb^+^ healthy controls (P<0.05) and HBV carriers or inactive HBsAg carriers (P<0.01). No significant difference was identified among the other groups (P>0.05; Fig. 4).

### Correlation of TFH cells, CD19^+^ B cells and IL-21 level with the clinical indicators of CHB patients

The levels of HBV viral load, alanine aminotransferase (ALT) and aspartate aminotransferase (AST) of the CHB patients were 5.7±2.8 (log10 copies/ml), 102±227.1 U/l and 88±152.2 U/l, respectively. No significant correlation was identifed among the percentage of TFH cells, CD19^+^ B cells, IL-21 level, HBV viral load level, ALT and AST (P>0.05). There were 24 HBeAg^−^ and 18 HBeAg^+^ cases among 42 patients with CHB. No significant differences were identified in the percentage of TFH cells and the expression level of CD40L molecules between the HBeAg^−^ and HBeAg^+^ groups (P>0.05). The IL-21 expression level was 402.2±156.7 ng/l in the HBeAg^−^ group and 344.5±261.2 ng/l in the HBeAg^+^ group. No significant difference was identified between the two groups (P>0.05; Table I).

### Correlation between the TFH cells and B cells in patients with CHB

The percentage of TFH cells in CD4^+^ T cells was 26.1±13.3% in the 42 patients with CHB. The level of CD40L expression in the TFH cells was 54.2±27.9%. The percentage of CD19^+^ B cells in peripheral blood mononuclear cells was 11.7±7.8%. The level of CD40 molecular expression in CD19^+^ B cells was 94.3±5.4%. A positive correlation was observed between CD40L expression in TFH cells and CD40 expression in CD19^+^ B cells (r=0.391, P=0.011; Fig. 5). No correlation was observed between the percentage of TFH cells and CD19^+^ B cells (r=0.172, P=0.276).

## Discussion

T helper cells are required for B cell-mediated humoural immune responses. Previous studies have shown that Th2 cells play a key role in aiding B cell responses; however, TFH cells have been recently recognised as the major subset that aids B cell responses. A number of studies have reported on the role of TFH cells in immune-related disease; however, few studies have described their role in chronic HBV infection (7,10). Feng *et al*(11) identified that TFH cells are involved in the immune response in HBV infection and their increase in number reflects the activation of the immune response. The results of the present study revealed that the percentage of TFH cells increased in patients with chronic HBV infection compared with healthy subjects. The percentage of TFH cells in the CHB patients was higher than that in the chronic HBV carriers and inactive HBsAg carriers. These results suggest that the elevation of TFH cells in CHB patients is associated with the activation of anti-HBV immune responses and are consistent with the study by Feng *et al*. Some studies showed that the expression of CXCR5 in the activation of T cells is transient and rare, and is only persistently expressed in TFH cells (6,12). Therefore, the effect of CD4^+^ T cell activation on the changes of TFH during HBV infection may be excluded.

The high expression level of CD40L in TFH cells binding to CD40 in B cells plays an important role in stimulating B cell proliferation, differentiation and immunoglobulin class switching (13). Wu and Wen demonstrated that the percentage of CD19^+^ B cells in CHB atients was significantly higher than in healthy controls (14). In the present study, compared with HBsAb^−^ healthy controls, the percentage of CD19^+^ B cells was elevated and the percentage of CD40 molecules on the surface of CD19^+^ B cells decreased in patients with CHB. The percentage of CD40L molecules on the surface of TFH cells in CHB patients was significantly elevated. There was a positive correlation between the level of CD40L expression in TFH cells and CD40 expression in CD19^+^ B cells. These results suggest that the activation of B lymphocytes in patients with CHB may be involved in the dysfunction of the humoural immune response of CHB.

TFH cells produce numerous cytokines, including IL-4, -10, -17 and -21, among which the most important is IL-21. IL-21 is the major cytokine of TFH cells and also a key factor affecting the formation of germinal centres. IL-21 is also known as TFH cell helper factor (15). Hu *et al*(16) reported that IL-21 promotes B-cell proliferation and HBeAg^−^ IgG secretion in CHB patients and may play a role in the serological conversion of HBeAg to HBeAb. The results of the current study revealed that the IL-21 level decreased in the plasma of HBV and inactive HBsAg carriers; however, it increased in CHB patients. These results suggest that IL-21 expression may be correlated with the immune response against HBV infection, similar to the alteration of TFH cells. There was no clear difference between the IL-21 levels of the HBeAg^+^ and HBeAg^−^ patients. No significant correlation was identified between IL-21 expression and the levels of HBV DNA, ALT and AST, which differs from the results of the study by Feng *et al*(11). The cause of these discrepancies may be related to patient selection and the research methods used.

In addition to promoting the differentiation of TFH cells and stimulating B cell proliferation, IL-21 also promotes the generation of interferon (IFN)-γ and counteracts regulatory T cell-mediated immune suppression. Additionally, it enhances CD8^+^ T cell and natural killer (NK) cell cytotoxicity (17). A previous study demonstrated that IL-21 participates in the immune response of viral infection clearance in acute HBV infection. However, this phenomenon is not observed in CHB patients (18). Decreased IL-21 production may block the key function of CD8^+^ T cells and B cell response, influencing the immune response against HBV. The results of the current study revealed that the IL-21 level decreased in chronic HBV carriers and inactive HBsAg^+^ carriers and the percentage of TFH cells was significantly elevated. These results suggest that the activity of TFH cells may decrease in chronic HBV and inactive HBsAg^+^ carriers. The level of IL-21 and TFH cells synchronously increased in the CHB patients. Yi *et al*(19) reported that IL-21 and IL-21-producing cells (TFH cells) are important in generating and maintaining multi-functional CD8^+^ T cells to clear the viral infection. The TFH cell number and/or abnormal function, as well as IL-21 expression deficiency, may be closely associated with the chronicity of hepatitis B virus infection. However, several studies have demonstrated that Th17 cells, CD8^+^ T cells and NK T cells also produce amounts of IL-21, in addition to TFH cells (20). The effect of these cells on the expression level of IL-21 requires further research.

In conclusion, the results of the present study suggest that the abnormal expression of TFH cells and IL-21 is related to the dysfunction of the immune response during chronic HBV infection. The interaction of CD19^+^ B cells with TFH cells via their CD40 and CD40L molecules may be significant in this process.

## Figures and Tables

**Figure 1.** Flow cytometry analysis of TFH cells. (A) Analysis of lymphocyte cells. R1, lymphocyte cell population; (B) analysis of the CD4^+^ T cell subset. R2, CD4^+^ T cell subset population; (C) analysis of TFH cells (isotype control); (D) analysis of TFH cells (CD4^+^ CXCR5^+^ cells). TFH, T follicular helper; CXCR5, CXC chemokine receptor 5.

**Figure 2.** Comparison of the expression of TFH cells and their surface CD40L molecule. 1, HBsAb^−^ healthy controls; 2, HBsAb^+^ healthy controls; 3, chronic HBV carriers; 4, inactive HBsAg carriers and 5, chronic hepatitis B. (A) Percentage of TFH cells. P<0.01, between groups 1, 2 and 3, 4, 5. (B) Percentage of CD40L. P<0.01, between groups 1,2 and 3, 4, 5. (C) Coexpression of CXCR5^+^ CD40L^+^ cells. P<0.01, between groups 1, 2 and 3, 4, 5. TFH, T follicular helper; HBsAb, hepatitis B surface antibody; HBV, hepatitis B virus; HBsAg, hepatitis B surface antigen; CXCR5, CXC chemokine receptor 5.

**Figure 3.** Comparison of the expression of CD19^+^ B cells and their surface CD40 molecule. 1, HBsAb^−^ healthy controls; 2, HBsAb^+^ healthy controls; 3, chronic HBV carriers; 4, inactive HBsAg carriers and 5, chronic hepatitis B. (A) Percentage of CD19^+^ B cells. P<0.05, between groups 3, 4 and 5. (B) Percentage of CD40. P<0.01, between groups 1 and 3, 4 and 5. HBsAb, hepatitis B surface antibody; HBV, heptitis B virus; HBsAg, hepatitis B surface antigen; PBMC, peripheral blood mononuclear cells.

**Figure 4.** Comparison of IL-21 expression levels. 1, HBsAb^−^ healthy controls; 2, HBsAb^+^ healthy controls; 3, chronic HBV carriers; 4, inactive HBsAg carriers and 5, chronic hepatitis B. P<0.05, between the levels of IL-21 in groups 1 and 3; 2 and 4, 5; P<0.01, between the levels of IL-21 in groups 1 and 4; 3, 4 and 5. IL, interleukin; HBsAb, hepatitis B surface antibody; HBV, hepatitis B virus; HBsAg, hepatitis B surface antigen.

**Figure 5.** Correlation between the levels of CD40L and CD40 expression. TFH, T follicular helper.

**Table I.** Comparison of the levels of TFH and IL-21 between the HBeAg^−^ and HBeAg^+^ groups.

Group	n	TFH cell (%)	CD40L (%)	IL-21 (ng/l)
HBeAg^−^	24	25.2±15.2	51.4±18.0	402.2±156.7
HBeAg^+^	18	28.0±12.0^a^	54.8±31.5^a^	344.5±261.2^a^

a P>0.05, compared with the HBeAg^+^ group. TFH, T follicular helper; IL, interleukin; HBeAg, hepatitis B e-antigen.
